# Innovative Research on Teaching Method of Taekwondo in College Elective Courses under the Background of Big Data

**DOI:** 10.1155/2022/2329952

**Published:** 2022-01-05

**Authors:** Yahui Chang, Su Meng, Hong Chao

**Affiliations:** ^1^School of Physical Education, Shanxi University, Taiyuan, China; ^2^School of Department of PE, Dankook University, Yongin-si, Republic of Korea

## Abstract

In the new stage of the new century, a new technological revolution is coming quietly. This revolution is represented by “data.” The application of “big data (B D A)” technology is causing changes in all walks of life, and the use of “B D A research methods” in the education field will inevitably become a trend. The purpose of this article is an innovative research on the teaching methods of Taekwondo based on the background of B D A in a college elective course. This paper first introduces the core technology of the database by summarizing the basic theory of the database. Based on the current situation of elective Taekwondo teaching in contemporary universities, analyze the current problems and deficiencies and conduct innovative research on college elective Taekwondo teaching methods combined with Beidou technology. This paper systematically expounds the practical connection, method innovation, and implementation path between BDA technology and college elective Taekwondo teaching methods and compares the traditional Taekwondo teaching methods based on BDA technology. Experimental research shows that compared with traditional Taekwondo teaching methods, the performance of university Taekwondo teaching based on data mining (D M I) in the context of B D A is more than 20% higher, which fully reflects its feasibility and the innovation of traditional Taekwondo teaching methods needs to be solved urgently.

## 1. Introduction

With the rapid development of Taekwondo, new curriculum reforms, and advances in technology, the requirements for Taekwondo teaching are getting higher and higher [1, 2]. Now, Taekwondo teaching still faces some problems: for example, the level of Taekwondo coaches is uneven, lack of innovation ability, outdated teaching methods, and lack of venue facilities [3, 4]. Combining B D A technology is one of the very important ways to innovate the teaching method of Taekwondo in college elective courses [5, 6].

In the research on the innovation of Taekwondo teaching methods, many scholars have made good achievements. For example, Junyi believes that Taekwondo theory learning and practical teaching should be emphasized in the teaching process [7, 8]. Bian Wenhong started with the basic connotation of happy physical education. Teachers teach happily, let students learn in a pleasant atmosphere, and cultivate their initiative and creativity [9, 10]. Students learn in a happy, relaxed, and harmonious environment, rather than being forced to accept, so as to cultivate their lifelong awareness of sports [11, 12].

The purpose of this article is to promote the development of higher education in our country. The purpose of this article is to conduct innovative research on the Taekwondo teaching methods of college elective courses based on B D A technology. By combining the traditional Taekwondo teaching methods with the Taekwondo teaching of college elective courses based on B D A technology, the methods are compared and analyzed to judge the feasibility of the innovation of the teaching method of Taekwondo as an elective course in colleges and universities under the background of B D A.

## 2. The Application Research of University Elective Course Taekwondo Teaching System Based on Big Data

### 2.1. Background Connotation of B D A

In the context of the information age, with the rise of new media such as digital terminals, cloud services, Weibo, and WeChat, information data is also showing an exponential growth trend. At present, there is no unified definition of B D A, but the academic circles basically believe that it mainly refers to software and hardware tools and data related to the perception, collection, processing, management, and service of the assembly. It has the characteristics of low value density, diversity, scale, and high speed and can be divided into structured data, semistructured data, and unstructured data [13].

### 2.2. Analysis of the Status Quo of Taekwondo Teaching in Colleges and Universities

Our country's physical education curriculum has always been in a passive state in actual teaching. Many schools' physical education classes are dominated by herding sheep. It is precisely because school leaders do not pay attention to physical education courses, which has caused some educators in our country to pay no attention to physical education courses. Taekwondo is part of the physical education curriculum, and it has also been ignored by teachers in teaching [14].

### 2.3. Analysis of Taekwondo Teaching Strategies for the Elective Course in Colleges and Universities with B D A Background

#### 2.3.1. Strengthen the Introduction of Full-Time Taekwondo Teachers and the Construction of Teaching Facilities

Teachers are one of the main groups in the entire teaching process. Adding new forces is an important measure to improve the overall level of Taekwondo teachers in colleges and universities. Teaching venues are an important factor that restricts teaching. Taekwondo is a sporting event that requires very high venue facilities. Therefore, the quality of venues and facilities affects the quality of teaching to some extent and limits the development of Taekwondo teaching.

#### 2.3.2. Optimize Teaching Courses

The curriculum setting must be set around the realization of the training goals, and the curriculum setting of the physical education major is the same. The reform of the physical education curriculum is a complex and cumbersome systematic program. It mainly includes several aspects. One is the reform of the curriculum content. The second is to optimize the curriculum structure. Optimizing the curriculum is a necessary condition for students to form a reasonable ability structure.

#### 2.3.3. Standardize Examination Standards, Etc.

Students' learning results can be reflected in test scores. Therefore, the test must be standardized. The test format can be diversified. A unified test standard can be formulated so that students can truly learn everything in the Taekwondo class. The courses are all for the sake of class. After the class is over, the content learned is also forgotten. After the Taekwondo course is completed, students should be able to take classes in elementary and middle schools or in a Taekwondo club. This is the purpose of setting up a Taekwondo course, which is also conducive to the future employment of students. It is more conducive to the development of school sports and national fitness.

### 2.4. Design of Taekwondo Teaching System for College Elective Course Based on D M I

#### 2.4.1. DMI Technology

The DMI process actually refers to using algorithms or rules to obtain hidden information from large amounts of data that can be achieved by various methods such as machine learning, mathematical analysis, and professional structure. WEB mining was developed by DMI and supports algorithms such as database techniques, classification, and clustering. If users of large websites are processing large datasets, multiple processors need to use parallel computing techniques to perform distributed processing.

#### 2.4.2. System Feasibility and Demand Analysis

*(1) Feasibility Analysis*. Nowadays, there are many kinds of learning resources on the Internet, and ordinary face-to-face classrooms cannot meet the learning needs of students for all kinds of knowledge. Currently on the Internet, new forms such as video courses such as microclasses are emerging in an endless stream. The curriculum resources are abundant but huge, and students cannot quickly find materials that suit them. In addition, the university elective course Taekwondo teaching lacks theoretical knowledge teaching, which requires the school to establish a resource database for the students of the school, so that students can choose appropriate teaching resources according to their own conditions and needs. Therefore, it is necessary to establish a system that can help students learn online and provide related services. The research of this project is to develop the university elective course Taekwondo teaching system based on D M I with the support of university campus network.

*(2) Demand Analysis*. The network-based network teaching system is aimed at three types of users: system administrators, network teachers, and students participating in online teaching. Teachers mainly need to lecture on the Internet platform, answer questions, take exams, review test papers, and evaluate teaching. For students, they also need to evaluate the teacher's teaching effectiveness. Therefore, the main task of the system is as follows: the system administrator uses the administrator account to manage the platform and is responsible for assigning specific user permissions and resources to users, so as to realize the allocation of teaching resources and the authorization of user functions. Teachers are responsible for the resource and authority settings of online courses, such as online courses, assignments, online questions, and test evaluations.. Teacher accounts can be used to generate course resources, manage the classroom right to participate, implement online teaching, online work management, online Q and A, etc., and the purpose of evaluating and evaluating the students' performance. Students are responsible for attending classes, taking exams, taking questions, using the student account to obtain course applications, asking questions, and completing course assessments during the study process.

#### 2.4.3. Overall System Design

The university Taekwondo teaching system based on B D A allows students to use the self-test platform provided by the system to understand the mastery of theoretical knowledge in time and participate in the course of the course in time.

*(1) Detailed Design of Online Course Modules*. The online course module is mainly to display the course title of the course on the homepage. When you log in to the detailed interface, there is a detailed introduction of the fine course such as pictures. At the same time, both the administrator and the teacher can maintain the course. When the administrator or teacher adds a course, find out whether there is corresponding course information. If not, create the course.

*(2) Database Design*. The design structure of course schedule is shown in Table 1.

### 2.5. Application of Collaborative Filtering Algorithm in Teaching Resource Recommendation

When a user A needs personalized recommendation, you can first find a user group G similar to his interest and then recommend what G likes and A has not heard of to A, which is the user-based system filtering algorithm.

Pearson coefficient is a similarity calculation method based on correlation coefficient. It needs to find the common score of the users in order to make accurate calculation results. *U* is the set of users who rated item *i* and item *j*, and the Pearson correlation coefficient formula is as follows:

(1) $$\begin{array}{c} \text{sim}\left(i,j\right)=\frac{\sum_{u\in U}\left(R_{u,i}-\bar{R_{i}}\right)\left(R_{u,j}-\bar{R_{j}}\right)}{\sqrt{{\left(\sum_{u\in U}R_{u.i}-\bar{R_{i}}\right)}^{2}}\sqrt{{\left(\sum_{u\in U}R_{u.j}-\bar{R_{j}}\right)}^{2}}}. \end{array}$$

Among them,  *R*_*u*,*i*_ is the rating of user *i* on item *j*, and *R*_*i*_ is the rating of item set *U* on the same item.

The implementation of collaborative filtering recommendation system relies on user ratings and other behaviors; so, it is a good idea to use clustering methods to divide the population into several categories. This paper intends to introduce a hybrid algorithm based on the combination of clustering algorithm and collaborative filtering algorithm to solve the problems in recommendation, increase recommendation efficiency, and increase recommendation quality. The algorithm is as follows:

(2) $$\begin{array}{c} \text{sim}\left(u_{1},u_{2}\right)=1-\frac{\sqrt{\sum_{u\in U}{\left(r_{u_{1},i}-r_{u_{2},i}\right)}^{2}}}{\text{commonItems}}. \end{array}$$

## 3. Taekwondo Teaching Experimental Research in College Elective Courses under the Background of Big Data

### 3.1. Subjects

1. In order to make the experimental data of this article more scientific and effective, this experiment conducted indepth interviews with students who have taken the Taekwondo course and teachers who teach Taekwondo through face-to-face interviews with colleges and universities in a certain place. The course conducts experimental research and analysis on the problems existing in the teaching content
2. In order to further study the Taekwondo teaching method of college elective courses in the background of B D A, this experiment compares the traditional Taekwondo teaching method with the college elective course teaching method based on B D A. The Taekwondo teaching system of D M I is indepth research. This study uses a questionnaire survey method. The surveyed students are all juniors and above. The juniors have completed most of the courses, which can better ensure the validity of the data obtained from the questionnaire survey

### 3.2. Research Methods

#### 3.2.1. Questionnaire Survey Method

This article asks relevant experts to set up targeted questionnaires and uses a semiclosed method to survey college students, the purpose of which is to promote relevant students to fill in correctly.

#### 3.2.2. Field Research Method

This paper analyzes the data obtained from conducting face-to-face interviews and data collection with teachers and students in school Taekwondo courses somewhere. These data provide theoretical support not only for the topic selection in this paper but also for the last article. The results of this study provide a reliable reference.

#### 3.2.3. Mathematical Statistics

Use relevant software to sort out and analyze the final research results.

## 4. Taekwondo Teaching Experiment Analysis of College Elective Courses under the Background of Big Data

### 4.1. Analysis of Problems in the Content of Taekwondo Course

#### 4.1.1. Analysis of Teachers' Teaching Ability

The teacher's teaching method will directly affect the students' interest in the course. The teacher's teaching ability is his ability to engage in teaching work, and it has a significant effect on the adaptation of teaching development and the improvement of quality. The satisfaction of students with the teacher's teaching ability is shown in Table 2.

It can be seen from Figure 1 that more than 95% of the students are satisfied with the teacher's teaching ability. Therefore, on the whole, the teacher's teaching ability is widely recognized by the students, but there are still a small number of students who think that the teacher's ability is not outstanding enough. It also needs continuous improvement.

#### 4.1.2. Analysis of Problems in Teachers' Teaching Methods

The quality of teaching methods will directly affect students' interest in learning. The problems in teachers' teaching methods are shown in Table 3.

It can be seen from Figure 2 that the main problems in the teaching method are the single teaching method, the lack of student practice, and insufficient teaching hours. The side reflects that the Taekwondo teaching method of the elective courses in universities in our country is too monotonous and boring, and the teaching method of Taekwondo is too boring. Innovation needs to be solved urgently.

### 4.2. Taekwondo Teaching System Analysis Based on D M I

#### 4.2.1. Comparative Analysis of Taekwondo Teaching

In order to make the data in this article more scientific and effective, this experiment compares the traditional Taekwondo teaching method with the Taekwondo teaching system based on D M I in college elective courses. The experimental data obtained are shown in Table 4.

It can be seen from Figure 3 that compared with the traditional teaching method of Taekwondo, the university elective teaching system of Taekwondo based on D M I is more excellent in all aspects of Taekwondo teaching, especially in the area of curriculum resources, which is more efficient than traditional teaching methods. 20% massive data under the background of B D A can more effectively make up for the shortcomings of traditional Taekwondo teaching content.

#### 4.2.2. Performance Analysis of University Taekwondo Teaching System Based on D M I

In order to carry out experimental research and analysis of the university Taekwondo teaching system based on D M I designed this time, this experiment conducted an analysis and research on the university Taekwondo teaching system based on D M I through interviews with relevant teachers and students. The experimental data is shown in Table 5.

It can be seen from Figure 4 that most of the Taekwondo professional teachers and students are satisfied with the Taekwondo teaching system based on D M I, especially in the area of convenience. The performance of the Taekwondo teaching system based on D M I is higher, which fully reflects the design based on this time. The feasibility of Taekwondo teaching system based on D M I in college elective courses.

## 5. Conclusion

As a kind of educational practice activity, the realization degree and implementation effect depends on the science and modernity of methods and means. Only in the face of the new changes in the situation and tasks brought about by technological progress and technological innovation can the innovative teaching methods of Taekwondo make the Taekwondo teaching more attractive and full of new vitality. Today, BDA technology has changed the teaching model that has lasted for thousands of years. Taekwondo teaching should also stand at the forefront of the BDA era, keenly perceive the more convenient, efficient, and personalized teaching methods brought by BDA, have an indepth understanding of the innovation of teaching thinking caused by BDA, and actively choose to cooperate with BDA. The integration of data will raise the improvement of Taekwondo teaching methods to a new level. Experimental research shows that compared with traditional Taekwondo teaching methods, the performance of university Taekwondo teaching based on data mining (D M I) in the context of B D A is more than 20% higher, which fully reflects its feasibility and the innovation of traditional Taekwondo teaching methods needs to be solved urgently.

## Figures and Tables

**Figure 1:** Analysis of teachers' teaching ability.

**Figure 2:** Analysis of problems existing in the teaching method of level teacher.

**Figure 3:** Comparative analysis of Taekwondo teaching.

**Figure 4:** Performance analysis of Taekwondo teaching system in colleges and universities based on D M I.

**Table 1:** Course.

Field name	Field type	Primary key	Is it empty	Definition
Id	Int	Pri	No	Auto_increment
course_number	Varchar (20)	No	Yes	
Title	Varchar (30)	No	No	
Teacher	Varchar (20)	No	No	
Info	Varchar (500)	No	Yes	
Course_studentno	Varchar (20)	No	Yes	

Table description: the id number of the id course is unique. It uses the int type and is the primary key of the table. It cannot be empty. Auto_increment is the realization of automatic growth.

**Table 2:** Analysis of teachers' teaching ability.

	Very satisfied	Satisfaction	Not so satisfied	Dissatisfied
Man	45	92	5	2
Woman	41	90	6	0

**Table 3:** Analysis of problems existing in the teaching method of level teacher.

	Man	Woman
Rigid teaching methods	37	34
Single teaching form	75	50
Students practice too little	82	80
Insufficient teaching hours	78	103
No problem	5	2

**Table 4:** Comparative analysis of Taekwondo teaching.

	Course resources	Teaching method	Teaching content	Standard test
D M I	75.2%	68.4%	69.7%	71.5%
Traditional	55.4%	59.7%	67.5%	63.2%

**Table 5:** Performance analysis of Taekwondo teaching system in colleges and universities based on D M I.

	Safety	Convenience	Robustness	Scalability
Teacher	12	25	8	9
Student	15	31	12	13

## Data Availability

The data underlying the results presented in the study are available within the manuscript.
